# Meta-Resolve of Risk Factors for Nosocomial Infection in Patients Undergoing Thoracic Surgery

This article has been retracted.

**DOI:** 10.1155/2022/2836014

**Published:** 2022-09-29

**Authors:** Junjian Chen, Wanyi Zhang, Deshu Yang

**Affiliations:** Department of Cardiothoracic Surgery, Chongqing Emergency Medical Center, Chongqing University Central Hospital, Chongqing, China

## Abstract

As we all know, various complications may occur after surgery, and postoperative bleeding and infection are the most common in clinical practice. Postoperative infection mainly manifests as abdominal abscess, peritonitis, and fungal infection. Thoracic surgery is a very common clinical operation. It can directly deal with the relevant lesions, so a better curative effect can usually be obtained. However, patients undergoing thoracic surgery are generally more severely ill, with low immune resistance, long duration, and complicated surgical treatment process. Therefore, the probability of nosocomial infection is high, and there are many risk factors for infection. After the occurrence of HAI, it not only increases the suffering and economic burden of patients and the workload of medical staff but also prolongs the hospitalization time of patients, reduces the turnover rate of hospital beds, causes unnecessary economic losses, and affects the social and economic benefits of hospitals. Based on this, this paper proposes to analyze the risk factors of nosocomial infection in patients undergoing thoracic surgery, so as to provide a reference for the prevention or control of nosocomial infection. This paper analyzes the actual situation of nosocomial infection in a city hospital and then uses meta-analysis to determine the factors of nosocomial infection from the perspective of relevant research literature. Meta-analysis results show that patients older than 60 years have twice the risk of postoperative infection compared with patients younger than 60 years.

## 1. Introduction

As an important medical specialty, thoracic surgery has been established for more than 100 years and has made great contributions to patients and society. Thoracic surgery specifically examines, diagnoses, and treats pathological changes in the thoracic organs such as the lungs, esophagus, and mediastinum. At present, the surgical treatment methods for thoracic surgery mainly include two categories: thoracotomy and thoracoscopic surgery. Thoracotomy, with a large incision size, mainly includes pleurectomy, and resections for single wedge, multiple wedges, lung segments, sleeve lobes, lobes, and whole lungs. Thoracic surgery is an important part of the operating department of the hospital, and it is an important area for the treatment and rescue of thoracic surgery diseases and critically ill patients. According to reports, the prevalence of nosocomial infection in thoracic surgery is on the rise, and life-threatening infections often occur, which causes huge economic losses and mental distress to patients.

Thoracic surgery mainly involves surgery for pleural cavity, lung, esophagus, and mediastinal masses. Due to the influence of anesthesia, the trauma is often large, the operation time is long, and there are many postoperative complications, including intraoperative respiratory and circulatory dysfunction, intraoperative and postoperative stress response, and decreased immune function. According to the latest reports, perioperative pulmonary rehabilitation in thoracic surgery is not only beneficial to reduce pulmonary complications but also is closely related to the overall recovery and increased activity of patients after surgery. Pulmonary rehabilitation training also emphasizes the rational application of antibiotics and the effective control of infection. Unreasonable use of antibacterial drugs not only fails to achieve the expected effect but also may cause adverse drug reactions and increase the medical cost for patients. Therefore, it is of great significance to rationally apply antibiotics to prevent and control the infection of patients in the perioperative period of thoracic surgery, so as to promote postoperative recovery of surgical patients and relieve the pain of patients.

In this paper, patients in thoracic surgery in a city hospital are used as the survey samples to analyze the nosocomial infection of patients in thoracic surgery in reality, and the probability of infection in thoracic surgery in this hospital can be obtained by calculation. The actual hospital survey shows that the incidence of nosocomial infection in thoracic surgery patients in this hospital is 8.5%, and the incidence of cases is 9%. It also roughly lists the common infection sites in nosocomial infections, as well as the infection situation of the number of doctors' operations, so as to better provide relevant protection suggestions to relevant workers. Then, meta-analysis is used to define the nosocomial infection factors from the perspective of related research literature. In conclusion, according to the meta-analysis results, several factors, such as male gender, general anesthesia, age >60 years, use of antibiotics, and operation time >4 hours, are risk factors for infection after thoracic surgery.

## 2. Related Work

The analysis of the current situation of nosocomial infection in patients undergoing thoracic surgery, and the related research for the purpose of preventing and controlling nosocomial infection has also become the focus of scholars from all over the world. Xue evaluated risk factors for IRS in patients with complex internal carotid aneurysms undergoing open microsurgery and bypass surgery, the results were analyzed for twenty patients (38 ± 12 years old). Quantitative digital subtraction angiography was found to be useful for the preoperative assessment of cerebral blood volume. This preoperative assessment can determine the appropriate treatment plan to prevent postoperative IRS [1]. Zhang conducted a comprehensive search of PubMed, EMbase, CNKI, and Wanfang databases to examine risk factors for postoperative infection in Chinese lung cancer patients. Meta-analysis revealed that older age, male gender, diabetes, smoking, squamous cell carcinoma, lung disease, duration of mechanical ventilation, and duration of surgery were associated with an increased risk of postoperative infection. In addition, prophylactic antibiotic therapy was associated with a decreased risk of postoperative infection [2]. Wang aimed to study the incidence of sepsis-induced cardiomyopathy (SICM) in patients undergoing general thoracic surgery and the risk factors and management strategies for this complication. Wang conducted a retrospective analysis of clinical data from 163 patients with postoperative sepsis. The results showed that the overall incidence of postoperative SICM was 53.99%. Multiple logistic regression analysis showed that stroke volume and CRP were independent predictors of mortality in patients with postoperative sepsis [3]. The study by Suleiman reported on nasal carriage of *S*. *aureus* and methicillin-resistant *S*. *aureus* (MRSA) in hospital and non-hospital centers. Although not all infections are causally associated with persistent carriage of *S*. *aureus* or MRSA, there are sufficient data to suggest that once immunity is compromised or immune defenses are broken, MRSA carriage may become a host for the development of subsequent infections [4]. The quality and quantity of the abovementioned related studies are limited, and more high-quality studies are needed to verify the abovementioned results.

In the study of thoracic surgery-related operations and related nosocomial infection factors, Zhou compared the proportion of patients with nasal infections among confirmed patients and the distribution of health care workers with nasal infections. The conclusion is that: at the beginning of the outbreak, the proportion of COVID-19 patients with nasal infections was 44%. Patients, who visit health care facilities, need good personal protection. Health care workers need to raise awareness of the disease to protect themselves and their patients [5]. Ambrogi started a program to perform video-assisted thoracoscopic surgery (VATS) for pulmonary metastasectomy under nonintubated local anesthesia. In this study, they investigated the effectiveness and long-term outcomes of this combined surgical anesthesia technique. VATS pulmonary metastasectomy under nonintubated local anesthesia is safe for selected patients with the oligometastatic disease and offers significant advantages in terms of overall operative time, length of stay, and economic cost. Morbidity is low but not significant, and long-term outcomes are similar [6]. Ismail reported his experience with U-VATS for the treatment of pleural effusion. The results showed that the mean age of the patients was (57.26 ± 18.29) years and 54.3% were male. In 85.7% of cases, pulmonary edema was associated with complex pneumonic pleural effusions, and only 5 cases were the result of surgery. Of these, 23 required chest tube insertion [7]. The abovementioned research results on the factors of nosocomial infection are mostly carried out from the perspective of a certain disease, the entry point is relatively small, and the research shown is more limited. There are few studies on nosocomial infection in thoracic surgery.

## 3. Exploring Methods of Nosocomial Infection

### 3.1. Concepts Related to Nosocomial Infection

Nosocomial infection refers to infection acquired by hospitalized patients, including infection during hospitalization and incubation period infection acquired in hospital. Infectious diseases contracted by hospital staff are also classified as nosocomial infections. Roughly speaking, the targets of nosocomial infection are inpatients, hospital staff, outpatients, emergency patients, visitors, family members of patients, and so on [8, 9]. It is often difficult to determine whether an infection came from a hospital. In fact, hospital-acquired infections primarily target hospitalized patients and hospital staff.

### 3.2. Main Sites of Nosocomial Infection in Patients Undergoing Thoracic Surgery

Respiratory infections: all patients undergoing thoracic surgery require endotracheal intubation for general anesthesia, which significantly impairs respiratory and circulatory physiology, and most thoracic surgeries involve the lungs and esophagus [10].

According to previous literature, the main site of nosocomial infection in cardiothoracic surgery is the respiratory tract, which accounts for about 65%. In thoracic surgery, there are many cancer patients and the elderly, and many patients with respiratory diseases. Respiratory function is damaged to a certain extent, cough is weak, sputum is difficult to discharge, and respiratory tract infection occurs [11, 12]. Patients with nosocomial infections also had the longest hospital stay for lower respiratory tract infections, with an average hospital stay of about 22 days.

Clinical diagnosis of urinary tract infection: the patient has urinary tract irritation symptoms such as frequent urination, urgency, dysuria, lower abdominal tenderness, tingling pain in the kidney area, and fever. And there is one of the following: (1) The urethral leukocytes are 5 or more high-power fields for men and 10 or more high-power fields for women. (2) Urinary tract infection is clinically diagnosed, or the response to antimicrobial therapy is confirmed as having a urinary tract infection [13].

The results of domestic and foreign literature studies showed that in Europe and the United States, urinary tract infections occupied the first place in nosocomial infections, followed by surgical site, skin and mucous membranes, and lower respiratory tract infections. In China, the order is given as follows: respiratory tract, urinary tract, surgical site, gastrointestinal tract, and so on [14].

Surgical site infection (SSI) is one of the most common postoperative complications. Many invasive procedures, most of which are severe, are likely to develop an infection due to large surgical wounds. It refers to a surgical infection that occurs in an incision or in a deep organ or surgical cavity. It includes: (1) Superficial incisional infections: infections limited to incised skin and subcutaneous tissue and occurring within 30 days of surgery. (2) Deep incisional infections: infections involving implants, including deep soft tissues and deep fasciae, such as artificial heart valves, artificial blood vessels, mechanical hearts, and artificial joints. (3) Organ (or cavity) infections: organ graft infections, including artificial blood vessels, mechanical hearts, or other implants, occurring within surgical-related infections (such as skin, subcutaneous, deep tendon, and so on) occurring within one year. Excluding infections of organs and cavities other than membranes and muscles such as joints [15, 16].

### 3.3. Thoracic Surgical Examination

If the patient is referred for thoracic surgery, the examination of the thoracic surgery includes physical examination, that is, the examination done by the doctor's sight, touch, percussion, hearing, and with the help of a stethoscope, sphygmomanometer, and other examination instruments. It is also called physical examination. The examinations done with the help of modern instruments include routine examinations such as electrocardiogram and chest X-ray, as well as routine blood tests, liver and kidney function, enzymatic examinations, physical and chemical examinations of pleural effusion, and bacteriological examinations of sputum and drainage fluid and so on [17]. Through these examinations, a basic understanding of most thoracic surgical diseases can be obtained, and a preliminary judgment of common thoracic surgical diseases can be made. In addition, it also includes examinations for special parts, such as aortic CT for aortic lesions, which is to understand the aorta. There are chest color ultrasound examinations for the presence or absence of pleural effusion, and PETCT for thoracic tumor surgery [18]. In addition, there are pathological examinations for excised tissue and puncture tissue. By perfecting the above related examinations, the specific condition of the patient can be roughly judged [19, 20]. As far as the modern medical industry is concerned, the determination of symptoms is closely related to medical images, and the quality of medical images seriously affects the diagnosis results of doctors.

Based on the abovementioned inspection requirements for medical images, several commonly used medical image enhancement techniques are briefly introduced here [21]. It helps to improve the accuracy of diagnosis [22].

Histogram equalization: the sharpness of the image is improved by changing the grayscale range of the image, and by increasing the number of pixels, the grayscale histogram of the image can be balanced within the range after transformation. Its processing steps are as follows.

First, the probability of occurrence of gray level in the input image is calculated, and the probability is expressed as K(ra).

The second is to calculate the distribution function.

(1) $$\begin{array}{c} F\left(ra\right)=\overset{a}{\underset{i=0}{\sum }}K\left(ri\right)\text{.} \end{array}$$

Among them,

(2) $$\begin{array}{c} a=0,1,2,\cdots ,m-1\text{.} \end{array}$$

The gray level *Ha*, *a*=1,2, ⋯, *E* − 1 of the transformed output image is obtained by calculation, where *E* represents the number of gray levels of the output image, and the calculation is given as follows:

(3) $$\begin{array}{c} Ha=INT\left[\left(H_{\max}-H_{\min}\right)+F\left(ra\right)+H_{\min}+0.5\right]\text{.} \end{array}$$

Among them, INT represents the rounding operation.

Then, on the basis of the previous step, the frequency of occurrence of gray levels is calculated.

Finally, the processed output image is obtained by adjusting *Ha* and *ra*.

Histogram equalization is designed to display better and more complete details for medical images related to bones, for over- and under-exposed images, and with less computation.

Mean filter method the mean filter method is based on the spatial domain and can perform simple smoothing on the original image:

(4) $$\begin{array}{c} A\left(m,n\right)=\overset{t}{\underset{f=-t}{\sum }}\overset{u}{\underset{s=-u}{\sum }}A\left(m-f,n-s\right)K\left(f,s\right). \end{array}$$

In the template, *M*, *n*=0,1,2, ⋯, *I* − 1. Among the mean filter and Gaussian low-pass filter, the most used is the mean average method, by taking 3 × 3 as an example.

(5) $$\begin{array}{c} R=\frac{1}{9}\times \left[\begin{array}{ccc} 1 & 1 & 1\\ 1 & 1 & 1\\ 1 & 1 & 1 \end{array}\right]. \end{array}$$

The template of the Gaussian filter is given as follows:

(6) $$\begin{array}{c} R=\frac{1}{16}\times \left[\begin{array}{ccc} 1 & 2 & 1\\ 2 & 4 & 2\\ 1 & 2 & 1 \end{array}\right]. \end{array}$$

In practical applications, the mean filtering method is simple to operate. Compared with other filtering methods, it has better processing speed and can effectively suppress surrounding noise [23, 24]. However, in the process of filtering, the useful details of the target are weakened with the filtering.

Median filtering: the advantages are that the amount of computation is less, the operation is easier, and in practical applications, noise isolation smoothing is better than average filtering, and the boundaries of the image can be better protected [25]. The disadvantage is that during the filtering process, the image losses local information such as thin lines [26].

(7) $$\begin{array}{c} A\left(i,j\right)=Median\left\{y\left(i-m,j-n\right),\left(m,n\right)\in \theta \right\}\text{.} \end{array}$$

Adaptive filtering: the purpose is to minimize the variance between the filtered image *M*(*i*, *j*) and the original image *N*(*i*, *j*) before being contaminated.

The variance expression equation is given as follows:

(8) $$\begin{array}{c} x^{2}=C\left[\left(N\left(i,j\right)-M\left(i,j\right)\right)\right]x^{2}. \end{array}$$

The advantage of this filter is that it has a wide range of applications and can well preserve the edge of the image, but it is weaker than other filtering methods in terms of calculation speed. Because of its large amount of computation, its execution capability is weak [27].

This section briefly introduces the methods of medical image enhancement processing and describes in detail the principles, scope of application, expressions, advantages, and disadvantages of various algorithms in filtering.

## 4. Survey Results of Nosocomial Infection in Thoracic Surgery

In order to investigate the factors of nosocomial infection in thoracic surgery, this experiment takes all patients admitted to thoracic surgery in a city hospital within two years as a data sample to investigate their infection. Then meta-analysis is used to analyze the actual influencing factors from the perspective of literature.

### 4.1. Investigating the Experimental Setup

#### 4.1.1. Correlation Calculation

The incidence of nosocomial infection Fr is given as follows:

(9) $$\begin{array}{c} Fr=\frac{Gr}{Zr}\times 100\%\text{.} \end{array}$$

Among them, Gr represents the number of nosocomial infections. Zr is the number of inpatients at the same time.

The probability of occurrence of nosocomial infection cases Lr is given as follows:

(10) $$\begin{array}{c} Lr=\frac{Ks}{Zr}\times 100\%\text{.} \end{array}$$

In the abovementioned equation, Ks represents the number of cases of infection in the hospital.

The occurrence density Ms of nosocomial infection is given as follows:

(11) $$\begin{array}{c} Ms=\frac{Gr}{Zc}\times 1000\%\text{.} \end{array}$$

Among them, Zc represents the number of bed-days of hospitalized patients during the same period.

The probability Ws of nosocomial infection for a certain risk index is given as follows:

(12) $$\begin{array}{c} Ws=\frac{Sb}{Sr}\times 100\%\text{.} \end{array}$$

In the abovementioned equation, Sb indicates the number of surgical site infections of a patient with a specified risk index for surgery, and Sr in it indicates the number of operations for a patient with a certain risk index for surgery.

The probability of occurrence of physician infection Yr is given as follows:

(13) $$\begin{array}{c} Yr=\frac{Bs}{Ts}\times 100\%\text{.} \end{array}$$

In the abovementioned equation, Bs represents the number of surgical site infections performed by physicians in patients with different risk index levels, and Ts is the number of cases performed by physicians in patients with different risk levels.

The average risk index Pu is given as follows:

(14) $$\begin{array}{c} Pu=\frac{Dw\times Sc}{Zc}\text{.} \end{array}$$

Among them, the risk index level is expressed as Dw, and Sc is the number of surgical cases. Zc represents the total number of surgical cases.

Physician-adjusted infection incidence rate Yz is as follows:

(15) $$\begin{array}{c} Yz=\frac{Yg}{Pw}\text{.} \end{array}$$

Among them, Yg represents the infection rate of physicians, and Pw represents the average risk level of physicians.

#### 4.1.2. Experimental Method

The experiments in this paper are carried out by sampling method. Under the condition that the patients were informed and agreed to participate in the experiment, a sample survey of thoracic surgery patients in this hospital is conducted. Patients, who had been infected before admission and those who did not agree to participate, were excluded from the above criteria. The details of the survey are shown in Table 1.

In order to ensure the accuracy of the data in this study, the main measures of quality control are: (1) Inclusion and diagnostic criteria are unified. (2) The thoracic surgeon is responsible for the clinical diagnosis of nosocomial infection, specimen collection, and inspection. (3) The data are collected by investigators, who need to go to the thoracic surgery ward every day. (4) According to the hospitalization number of the selected samples, the investigator conducts a secondary check of the information entered in the electronic medical record room to ensure the accuracy and completeness of the information in the survey form.

### 4.2. Investigation of Basic Infection in Hospitals

The number of noncompliant patients is excluded from this study, and the total number of patients included in the survey during the two years is 1219. The distribution of the number of infected people and the basic situation are shown in Table 2.

As shown in Table 2, the number of infected people in this hospital is 100, and the number of infections is 106. The infection rate in the second year is significantly higher than that in the first year. Its occurrence density is 4.1‰.

Figure 1 shows the incidence of infection and the incidence of cases of infection in the hospital within two years. The data comparison results showed that the hospital infection rate in the second year was significantly higher than that in the first year. As far as the infection rate was concerned, the infection rate in the first year was 8%, and it reached 9.1% in the second year, indicating that the infection rate of the hospital was between 8% and 9.1%, and the total infection probability was 8.55%. The number of infections shows that it is about 9% in the first year, 10% in the second year, and the total number of infections is 9%.

### 4.3. Nosocomial Infection Sites

Figure 2 shows the distribution of nosocomial infection sites for thoracic surgery patients at this hospital over a two-year period. Figure 2 (1) shows the distribution and composition of nosocomial infection sites in the first year of the survey, and the site with the highest infection rate is lower respiratory tract infection, which is more than 60%. The site with the lowest infection rate is a urinary tract infection, at just 2%. The site with the lowest infection rate is a urinary tract infection. The distribution of nosocomial infections in the second year shown in Figure 2 (2) is slightly different. Compared with the first year, the infection rate of the lower respiratory tract has decreased to 52%, but it is still the site with the highest infection rate. This is followed by upper respiratory tract infections at 18%. The lowest is pleural cavity infection, accounting for 5%. Urinary tract infections hardly occurred in the second year.

### 4.4. Infection Rate among Surgeons in Thoracic Surgery

From the perspective of the surgeons in the hospital, the infection rates and risk indices of different physicians are calculated, and the statistics are shown in Table 3. There are a total of 11 thoracic surgeons in the hospital, and the number of surgical cases varies greatly among physicians. By arranging it in descending order of the number of operations performed, it can be seen that physicians with less than 50 operations have almost no infection rate.

### 4.5. Antimicrobial Usage

Among the infected cases, more than 100 pathogenic strains are detected, mainly Gram-negative bacteria and Gram-positive cocci, accounting for more than 86% of all bacteria. It also includes a small number of fungi, which is without viral infections. Relevant statistics are made on the use of preoperative antibiotics and perioperative antibiotics, as shown in Figure 3.

As shown in Figure 3, patients' antimicrobial use over a two-year period is shown. In terms of preoperative medication use, the first-year medication rate was 67%, significantly higher than the second-year medication rate of 30%. According to the analysis of the drug use in each period shown in it, the medication before surgery is mainly a combination, and the perioperative period is mainly a double combination.

## 5. Meta-Resolve of Risk Factors for Nosocomial Infection

Through computer search, 6 databases of China National Journals Full-text Database (CNKI), China Biomedical Literature Database (CBM), VIP Database (VIP), Wanfang Database and foreign language database Pubmed, and the Cochrane Library and a manual search are used to comprehensively search the published research literature on risk factors for nosocomial infection in thoracic surgery. The languages are limited to Chinese and English. According to the literature screening process shown in Figure 4, 16 kinds of literature are finally obtained. According to the nosocomial infection factors actually collected by the abovementioned hospitals, from the perspective of relevant research literature, the risk factors of nosocomial infection are determined for the second time.

### 5.1. Different Genders

As shown in Figure 5, in the 16 eligible articles, 12 articles and 13 studies analyzed the effect of gender on nosocomial infection in patients undergoing thoracic surgery. There were a total of 2,212 surgical site infections, of which 716 were males, and 10,612 were controls, of which 5,279 were males. The heterogeneity test showed that there is little heterogeneity among the study results, *P*=0.2, *I*^2^ = 20.1%. Therefore, a meta-analysis using a fixed-effects model showed that the combined effect size OR = 0.9, 95% CI: 0.8–0.99, *P*=0.03, which indicating that gender is a risk factor for the prevention of nosocomial infection in thoracic surgery. The risk of postoperative wound infection is 0.9 times higher in male patients than in female patients. This may be related to women's thicker subcutaneous fat, which is more likely to be infected at the surgical wound.

### 5.2. Different Ages

As shown in Figure 6, 9 of the 16 included articles analyzed the effect of age on nosocomial infection in patients undergoing thoracic surgery. There were 3,374 cumulative surgical site infections, of which 735 were in patients over 60 years of age and 5,443 were in patients over 60 years of age. The results of the heterogeneity test showed that *P* < 0.01, *I*^2^ = 87.3%. Due to the large heterogeneity among the study results, a random-effects model was used for meta-analysis, which showed that the combined effect size was OR = 2, 95% CI: 1.7–23, *P* < 0.01. This suggests that patients over 60 years of age are a risk factor for nosocomial infection in thoracic surgery. Compared with patients under 60 years old, the risk of postoperative hospital infection is 2 times higher in patients 60 years and older.

### 5.3. Operation Time

As shown in Figure 7, 10 out of 16 eligible papers and 16 studies investigated the effect of operative time on nosocomial infection in patients undergoing thoracic surgery. There were a total of 1,683 surgical site infections, including 536 patients with an operation time >4 hours; 7,570 cases were controls, including 3,187 patients with an operation time >4 hours. The results of the heterogeneity test showed that *P* < 0.001, *I*^2^ = 90.4%. Due to the large heterogeneity between the study results, a random effect model was used for meta-analysis, which shows that the combined effect size OR = 2.6, 95% CI: 1.4–4.7, *P* < 0.001. It shows that the operation time >4 h is a risk factor for nosocomial infection after thoracic surgery, and for the operation time >4 h, the probability of nosocomial infection in patients undergoing thoracic surgery is 2.6 times higher than that when the operation time <4 h.

### 5.4. Use of Antimicrobials

As shown in Figure 8, 4 out of 16 eligible articles analyzed the impact of antimicrobial use on nosocomial infections in thoracic surgery patients. There were a total of 1,179 surgical site infections, of which 416 were medication patients, and 4,359 were controls, of which 1,232 were medication patients. The results of the qualitative test showed that there was little heterogeneity among the study results, *P*=0.11, *I*^2^ = 50%. Therefore, a meta-analysis using a fixed-effects model showed that the combined effect size OR = 1.6, 95% CI: 1.4–1.90, *P* < 0.01. This suggests that antimicrobial use is a risk factor for nosocomial infection after thoracic surgery and that in patients, who have undergone thoracic surgery, antimicrobial use is 1.6 times more likely than no antimicrobial use.

### 5.5. Influence of Anesthesia on Infection in Patients Undergoing Thoracic Surgery

As shown in Figure 9, there are three literature studies investigating the effect of the anesthesia method on nosocomial infection in patients undergoing thoracic surgery. There were a cumulative total of 4,630 surgical site infections, of which 486 were patients receiving general anesthesia, 211 were controls (regional anesthesia), and 78 were patients receiving general anesthesia. The results of the heterogeneity test showed that *P* < 0.001, *I*^2^ = 96.4%. Due to the large heterogeneity between the study results, a random effect model was used for meta-analysis, and it showed that the combined effect size OR = 0.4, 95% CI: 0.3–0.5, *P* < 0.001. This suggests that the use of general anesthesia is one of the factors of nosocomial infection after thoracic surgery. And it points out that, compared with the use of regional anesthesia, the risk of nosocomial infection in thoracic surgery patients with general anesthesia is 0.4 times that of regional anesthesia. This is inconsistent with routine organ intubation under general anesthesia, which is prone to respiratory infections. This may be related to the small sample size of the control group (local anesthesia group). Therefore, large samples and relevant multicenter studies are needed.

## 6. Conclusions

According to foreign reports, thoracic surgery causes great trauma to patients and is prone to nosocomial infection. The postoperative infection has a certain impact on cardiovascular and respiratory function. It has a significant impact on prognosis by increasing patient pain and treatment time. Therefore, it has important reference value for preventing and managing nosocomial infection and proposing corresponding remedial measures for an early understanding of the distribution and susceptibility factors of nosocomial infection. Based on this, this paper takes the patients of thoracic surgery in a city hospital as a sample to analyze the current distribution of nosocomial infection, which shows the importance of the analysis of risk factors for nosocomial infection. Then, from the perspective of relevant research literature, Meta-analysis is used to determine the current risk factors of post-operative nosocomial infection in patients, and further provide a reference for relevant workers. The results show that gender, anesthesia method, age, use of antibiotics, and operation time are risk factors for nosocomial infection after thoracic surgery. Of course, this study still has certain limitations. For example, the included type of literature are randomly selected, but they do not describe the specific method. Therefore, it may affect the objectivity of the experimental results.

## Figures and Tables

**Figure 1:** The infection rate and the number of infections in the hospital during the two years.

**Figure 2:** Distribution of infection sites in the thoracic surgery department of this hospital for two years.

**Figure 3:** Antimicrobial use.

**Figure 4:** Literature screening process.

**Figure 5:** Effect of gender on infection in thoracic surgery patients.

**Figure 6:** The effect of age on infection in thoracic surgery patients.

**Figure 7:** Effect of operative time on infection in patients undergoing thoracic surgery.

**Figure 8:** Effect of antimicrobial use on infection in thoracic surgery patients.

**Figure 9:** The effect of anesthesia on infection in patients undergoing thoracic surgery.

**Table 1:** Details of the survey.

Data classification	Details
1. Basic situation	Age, gender, admission diagnosis, discharge diagnosis, etc.
2. Surgical situation	Surgical incision healing, anesthesia, etc.
3. Nosocomial infection status of patients	Infection site, infection pathogen, etc.
4. Antimicrobial use	Dosage, time of use, etc.

**Table 2:** Nosocomial infection of patients undergoing thoracic surgery in a city hospital in two years.

Years	The first year	The second year	Total
Total number of operations	574	645	1219
Number of people infected	43	57	100
Infections	48	58	106
Inpatient bed days during the same period	11181	13934	25115
Average hospital stay	19.4	21.5	20.5
Occurrence density (‰)	4	4.2	4.1

**Table 3:** Occurrence probability of surgeons.

Surgeon	Number of surgeries	Number of infected cases	Infection rate	Hazard index			Adjusted infection rate
				0	1	2	
1	336	9	2.3	0.1	0.5	10	5.5
2	120	5	3.4	0	0.4	3.3	6.2
3	149	2	0.7	0.3	0	0	0.6
4	217	5	2.3	0	0.2	1	3
5	133	5	3.1	0	0.6	11.1	5.45
6	96	1	1.1	0.2	0	0	1.8
7	30	0	0	0	0	0	0
8	17	0	0	0	0	0	0
9	31	0	0	0	0	0	0
10	45	0	0	0	0	0	0
11	45	0	0	0	0	0	0

## Data Availability

Data sharing is not applicable to this article as no datasets were generated or analyzed during the current study.
